# Laticifer Identification, Rubber Characterization, Phenolic Content, and Antioxidant Activity of *Pergularia tomentosa* Latex Extract

**DOI:** 10.1155/2022/7158905

**Published:** 2022-07-20

**Authors:** Imen Lahmar, Mouhiba Ben Nasri-Ayachi, Karima Belghith

**Affiliations:** ^1^Laboratory of Ecosystems and Biodiversity in Arid Environment, Faculty of Sciences, Sfax, Tunisia; ^2^Laboratory of Plant Productivity and Environmental Restrictions, Faculty of Sciences El Manar, Tunisia; ^3^Laboratory of Plant Biotechnology Applied to Crop Improvement, Faculty of Sciences, Sfax, Tunisia

## Abstract

*Pergularia tomentosa* is a perennial twining herb widely spread out arid and semiarid Tunisian regions. It is searched for its richness in enzymes, secondary metabolites, antifungal activity, and milk-clotting activity. Traditional use implies the fresh latex in wounding heals. The present study was aimed at identifying laticifer distribution in *Pergularia tomentosa* stems, leaves, and petioles. In the present study, the identification of latex extract's components and its valorisation by estimation of phenolic content, flavonoids, and antioxidant activity are conducted. Anatomical structures proved the presence of laticifers in the aerial parts of *Pergularia tomentosa.* They are particularly observed along the pith and cortical parenchyma in stem, in leaf mesophyll, and in petiole phloem. Identified laticifers were characterized as nonarticulated. FTIR spectroscopy proves the presence of several functional groups in the latex and mainly the *cis-*1-4-isoprene monomer. Results suggested that *Pergularia tomentosa* latex contributes significantly as a source of phenol content (62.3 mg Eq GAE/g) and flavonoids (24.8 mg Eq QE/g). Scavenging free radicals of DPPH exhibited IC_50_ value of 12 *μ*g/ml. In conclusion, latex extracted from *Pergularia tomentosa* can be implied in industry as a natural rubber. It can be used, also, in medicine as a therapeutic agent.

## 1. Introduction

*Pergularia tomentosa* L. called as Bouhliba due to its latex belongs to Asclepiadaceae family and sub family of Asclepiadoideae. The species known by a lactiferous twinner presents follicles generally assembled together as twins and secreting at the slightest touch a sticky white fluid called latex [1]. In Tunisia, *P. tomentosa* represents the only species of the genus *Pergularia*. The plant is widespread in different countries of Mediterranean basin and Sahara (Algeria, Morocco, Egypt, Jordan, and Saudi Arabica) and often grown in Tunisia [2, 3]. In our country, traditional habit implies its integration to heal feet wounds, in tanning some clothes, and for depilatory procedure. Ethnopharmacological survey showed the implication of *Pergularia tomentosa* during the treatment of diarrhea, bronchitis, constipation, wound, and related injuries [4, 5]. Latex extracted from leaves was used to treat skin infections like *Tinea capitis* [6]. It is commonly administered as a poultice, abortifacient, laxative, and antihelmintic. Several important compounds screened in *P. tomentosa* like cardiotonic glycosides, uzarigenin, pergularoside, and *D*-glucopyranosylcalactin [7] correlate to this plant an important medicinal interest.

Castelblanque et al. [8] reported that around 12,500 plants belonging to 22 families secreting latex. This latex may contain enzymes, phenolic compounds, cardenolides, lipids, polysaccharides, triterpenes, alkaloids, and other components [9, 10]. The occurrence and amount of chemical compounds in each species led to an inconstant latex colour [11]. Thus, the appearance of this latex depended on the plant species-organ and can differ from clear to translucent [12]. In some family, it can be yellow, orange, brown, red, and colourless. In Apocynaceae, it is generally fluid and sticky with a milky-white colour [10]. *Pergularia tomentosa* latex was revealed as a stimulator agent on milk-clotting process [13].

A poisonous substance linked to lactucone and having a resinous character called aslepione was detected on the Asclepia latex [14]. The valorisation of *Pergularia tomentosa* as a source of natural latex bioinsecticide and the toxicity bioassay of its extract against *Locusta migratoria* showed that it can cause significant mortality by disturbing the respiratory rhythm and the hemocyte number [15]. In addition, due to their alkaloids localised in the aerial part of the plant, an important larvicidal potentiality was detected against the same insect [16]. Cardiotonic glycosides of *Pergularia tomentosa* were reported to have toxic effects against *Monacha obstructa*, land snail. This molluscidal activity can reach 96.6% [17].

Antifungal activity against *Fusarium oxysporum f.* sp. *Lycopersici*, a harmful pathogen of tomato vascular wilt, was recorded [18]. Indeed, this plant contained antibacterial, cytotoxic, and allelopathic compounds [6, 19, 20]. It was considered as antirheumatic and antitumor agent [21] and has hypoglyceaemic effects [22].

Latex is distributed throughout the plant in a special internal secretory system constituted by a series of elongated cells, called laticifers. By releasing their latex from laticifer cell combined to rubbers from parietal cytoplasm, latex-bearing plants construct a protective mechanism against herbivores and microorganisms as well as wound cicatrisation [10, 23]. A fast coagulation of latex revealed secretion efficiency to protect the plant [23, 24].

Latex production was combined to a distortion of cell contents leading, thus, a supply of required energy and an abundance of mitochondria, lipid bodies, starch grains, and osmiophilic structure transferred to the central vacuole [25]. The discontinuity of transverse cell walls associated to cell accumulation in protoplast is responsible of laticiferous cell creation [24, 26]. Latex secretion implies protoplasm degeneration, restriction of the cytoplasm, and fusion of small vacuoles with some vesicles into the central vacuole [27].

*Pergularia tomentosa* can be found in the arid lands of Tunisia, a main source of natural agent leading to hydrolysis of *κ*-casein and therefore milk-clotting procedure.

In order to valorise the species, the identification of cells excluding latex as well its chemical composition, phenolic content, and antioxidant activity of the secreted latex is very important. The present study identifies laticifers occurring in the stem, leaf, and petiole and even latex characterization.

## 2. Materials and Methods

### 2.1. Plant Material

Fresh plant of *Pergularia tomentosa* was collected in early morning in March from a Tunisian site belongs to subarid climate, Chebba. This site is a coastal town in the Tunisian Sahel located about sixty kilometers north of Sfax and about thirty kilometers south of Mahdia (Weather: 11°C, NW wind at 23 km/h, 63% humidity). Collection was done manually, and wearing plastic gloves was indispensible during the plant handling as a precaution from skin irritation due to the secreted latex at the slight touch. Plant material was authenticated by Pr. Mohamed Chaeib. Voucher specimen was deposit at the herbarium of the Laboratory of Ecosystems and Biodiversity in Arid Environment, Department of Biology, University of Sfax, LR18ES-29.

### 2.2. Extraction of Bioactive Compounds from Latex

At the moment of dripping stem extremities, latex was collected directly in sterile glass and kept at 4°C. The coagulable content identified as the percentage of dry rubber of latex was estimated according to the following formula [28]: dry rubber content (%) = (mass of dry coagulum/mass of latex) × 100. Following this method, latex sample will be used for Fourier transform infrared (FTIR) spectroscopy test.

By cutting stem apices, the latex was dropped swiftly and directly into the sterile glass tubes. The tubes already contained an equal volume of petroleum ether. The mixture was precipitated until the separation of petroleum ether layer. Aqueous layer containing pure latex were dried at 50°C for 48 h. The sample was then dissolved in 80% methanol with continuous agitation in shaker at 32°C and 140 rpm overnight to extract bioactive compounds from *Pergularia* latex [29]. Filtered solution considered as latex preparation was used for phenolic content and antioxidant activity tests.

### 2.3. Anatomical Study

After sampling, fresh leaves and stems were fixed in a Formalin-Acetic-Alcohol (FAA) mixture according to the Sass (1958) fixation procedure [30]. The fixed material was dehydrated by successive submersions in different solutions of distilled water and ethanol 95%. Serial transversal and longitudinal sections were made in a manual microtome (Leica RM2235). All sections were subsequently stained with aceto-carmin [31]. Anatomical observations were observed under a light Reichert LKB microscope and photographed with a digital camera (Olympus).

### 2.4. Fourier Transform Infrared (FTIR) Spectroscopy

Latex solution was pressed into pellets for the estimation of the Fourier transform infrared spectra with the scanned wave ranging from 4000 to 500 cm^−1^. Spectra were recorded on a PerkinElmer 1750 spectrophotometer equipped with a diamond attenuated total reflection (ATR) device.

### 2.5. Determination of Total Phenolic and Flavonoid Content

The total phenolic content was measured according to the Folin-Ciocalteu method based on the reduction of a phosphotungsten-phosphomolybdate complex [32]. 800 *𝜇*l of latex solution was added to 50 *𝜇*l of Folin-Ciocalteu reagent (2 N) and incubated for 3 min at room temperature. Then, 150 *𝜇*l of sodium carbonate solution was added. Absorbance was measured at 765 nm after 2 h of incubation in the dark. Gallic acid (GA) was used as a standard.

The total flavonoid content of the extracts was determined by the method of Lamaison and Carnat based on the formation of the complex flavonoid-aluminum [33]. The aliquot of latex solution (0.25 ml) was mixed with 0.5 ml of 2% aluminum chloride and incubated for 15 min. Absorbance was recorded at 430 nm. Quercetin was used as a standard.

### 2.6. Evaluation of Antioxidant Activity

The radical scavenging assay of methanolic extracts was measured as equivalent of hydrogen donor, according to the DPPH method [34]. 1,1-Diphenyl-2-picrylhydrazyl (DPPH) method was used for the determination of the antioxidant activity. 1 ml of freshly prepared DPPH solution (10−4 M) was added to 1 ml of latex solution at different concentrations (0.0625–2 mg/ml). Incubation was for 20 min at room temperature and dark. Absorbance was measured at 517 nm. The inhibition percent was calculated according to the following equation: radical scavenging effect (%) = [1–(optical absorbance of the latex solution/optical absorbance of the control)] × 100. BHT and *α*-tocopherol were used as positive control.

## 3. Results and Discussion

### 3.1. Morphological

In a warm period from spring to the beginning of autumn, the perennial herb shows greener and more compact with new shoots of leaves and stems. Leaves are opposite, cylindrical, and pubescent measuring about 10∗45 mm. Green-white petioles reached 22 mm of length for the adult plant. The young climbing stems of 3 mm of diameter twined around the old ones. Milky-white biological fluid named as latex was profusely exuded with a consistent dense at the slow injury of stem and leaf of *Pergularia tomentosa* (Figures 1(a), 1(b), 1(d), and 1(e)). All the aerial parts including stems, leaves, and petioles highlighted the latex exudation at the slight touch and a physical damage of the plant. The leaked latex was sticky and gives a small burning sensation when it is left on the skin for a long time. Stem showed saturated and fulfilled laticifers with a disposition in the pith and extremely in the cortex with a clear cylindrical arranging (Figure 1(c)).

### 3.2. Anatomical Study

Previous studies on laticifers focused on their distribution in plants and organs, their localisation, and identification of their types. In fact, they are considered as the main focus of herbivores and more exposed to microorganism attacks; the stems and leaves were the common organs of latex-bearing plant tissues [24]. Laticifer distribution patterns in plant species were very extent, and their types were various [35]. Their cell localisation depends on the vegetative organ and species genus [8, 36]. Nevertheless, there are few researches on anatomical structure at distribution on Asclepiadaceae (Asclepiades, Apocynaceae), and to our knowledge, there is no any anatomical previous research concerning laticifers in *Pergularia tomentosa*.

Our results revealed that, in stems, laticifers were located in the pith, in the collenchyma, and mainly in the cortical parenchyma (Figure 2). While, it was demonstrated that laticifers were identified in Apocynaceae stems and depending on the plant species, they could be observed in medullar radiuses, pericycle, phloem and pith. [37]. However, they can occur in the vascular tissue and cortical parenchyma in other species sections [26].

In leaves, laticifers were scattered in the mesophyll (spongy and palisade) and localised also in the central cylinder (Figure 3). Obtained results were in accordance to those found previously for other Asclepiadaceae [12, 27, 36, 38]. While in other study, secretory cells were found towards leaf extremities [26].

Cross section of *Pergularia* petiole showed two smaller and rounded lateral vascular bundles (Figures 3(c) and 3(d)). Laticifers located particularly in the phloem. In *Vinca sardoa* petiole, authors showed that laticifer cells were localised in the epidermis and the phloem parenchyma [39]. But in the case of *Euphorbia lathyris*, they were localised along the midrib of the petiole [8]. Laticiferous cell localisation can be considered as valuable criteria for taxonomical classification other than it differs within vegetative organs it is correlated to species nature.

Further studies described Asclepiadaceae laticifers as nonarticulate. They were dispersed in all parts of the plant from the pith to cortex and in vascular tissues and closely associated with the leaf phloem [26, 40]. Laticifers of *Vinca* [29], *Calotropis* [25], *Periploca* [28], and *Asclepias* [41] were identified as nonarticulated structures. Nevertheless, few species within Apocynaceae family were recognized as articulated anastomosing type like *Blepharodon bicuspidatum* belonging to Asclepiadoideae [24, 42]. Nonarticulate laticifers existed in families other than Asclepiadoideae, like *Asclepias speciosa* [41]; several species belonging to Euphorbiaceae, Moraceae, and Urticaceae have also single long laticifer cells branched without reconnection called nonarticulated laticifers [11].

Articulated laticifers have several interconnected simple and long cells, with intact or perforated transverse and lateral walls [36, 43]. Therefore, *Pergularia tomentosa* can be considered as nonarticulated laticifers.

### 3.3. FTIR Analysis of Latex

Latex sample was pressed into pellets for the estimation of the infrared spectra with the scanned wave ranging from 4000 to 500 cm^−1^. Spectra were recorded on a PerkinElmer Universal ATR Sampling Accessory (Figure 4). This method led to define the organic material functional groups and characterize their bonding information [44].

Several compound functional groups could be identified by Fourier transform infrared spectrum studies as alkenes, aromatic compounds, amines, carboxylic acids, amides, esters, alcohols, phenols, and nitro compounds [45]. The band 3349.28 cm^−1^ was probably related to the overlap of free O-H and N-H side groups descendant from amino group. Rubber oxidation may also be related. Vibration at 2067.15 cm^−1^ corresponds to carboxyl compound frequency, transition metal carboxyls, and nitrile compounds as expected phytocompound is identified. A vibrational mode characteristic from rubber main chain was defined at 1637.79 cm^−1^ related to C=C stretching. Bands at 1389.91 cm^−1^ and 1292.35 cm^−1^ indicate the presence of C-H bending, CH_2_ and CH_3_, respectively, corresponding to *cis-*1-4-isoprene monomer, while the peak at 591.28 cm^−1^, of low intensity, reveals predominantly C-C-C deformation vibrations. The mentioned functional groups present in the *Pergularia* latex are mainly correlated to the constituent mixture of sterols, fatty acids, proteins, sugars, gums, enzymes, etc. [18, 46].

### 3.4. Phenolic Content

A previous study highlighted the presence of phenolic compounds in stems, leaves, roots, and fruits of *Pergularia tomentosa* extracted following an increased gradient of polarity, with successively hexane, chloroform, ethyl acetate, and *n*-butanol [18]. Following the extraction method of active compounds from latex of *Pergularia tomentosa* described previously, the total phenolic and flavonoid contents of the latex extract were 62.3 mg Eq GAE/g latex and 24.8 mg Eq QE/g latex, respectively.

Furthermore, low contents in total phenolics and flavonoids were recorded in *Ficus carica* (50.2 mg GAE/g and 12.5 mg CE/g, respectively), *Euphorbia tirucalli* (10.5 mg GAE/g and 4.3 mg CE/g, respectively), and *Euphorbia dendroides* latex extracts (4.75 mg GAE/100 g and 1.46 mg RE/100 g FW, respectively) [29, 47].

Plants synthesize secondary metabolites like phenolic compounds and flavonoids occasionally for growth, essential physiological processes, and adaptive mechanism. Their production depended on the genotype and physiology of the species, environmental factors (temperature, sunlight exposure, dryness, and salinity), and growth stage of the plant. Abiotic and stress factors stimulate the plant to produce more of those compounds [48].

Consequently, they were implied in defence response to herbivore attacks and pathogenic microbial infection [49]. Moreover, researches proved that flavonoids possessed an important pharmacological interest and a significant antiproliferative effect [50]. In addition to phenolic, latex can contain carboxylated polysaccharides and lipophilic and hydrophilic substances as it was revealed in the case of *Tabernaemontana ventricosa.* Terpenoids, alkaloid neutral lipids, proteins, resin acids, acidic substances, mucilage, and pectin were also detected in latex of the vegetative organs [26].

### 3.5. Antioxidant Activity

Consuming natural antioxidants extracted from plants was recorded to boost the immunity system against danger system as cancer by their sweeping effect on the free radicals [51]. Antioxidant power can depend on many factors such as plant species and the reactivity and structure of the antioxidant. A strong positive correlation was established between phenolic content and antioxidant of *Pergularia tomentosa* fruits, stems, leaves, and root extracts [18].

In order to evaluate the antioxidant activity of *Pergularia tomentosa* latex, its ability to scavenge free DPPH was tested. The exhibited IC_50_ value was 12 *μ*g/ml. It corresponded to the extract concentration which is able to inhibit 50% of the free radicals. A low value indicates a high antioxidant activity. Among the latex samples recorded as source of natural antioxidants, *Ficus carica*, *Euphorbia tirucalli*, *and Euphorbia dendroides*, evaluated on the basis of their ability to scavenge DPPH, IC_50_ values were estimated, 13.6, 7.0, and 6.0 *μ*g/ml, respectively [29]. Moreover, the latex of *Pergularia tomentosa* can be considered as a promising source for several bioactive compound antioxidants. Other than its phenolic content, antioxidant ability of the latex extract might be related to the type of the solvent used for extraction and interaction between sample components [51, 52]. Also, phenolic content of the latex sample can have a different susceptibility toward free radicals of the selected solvent, they present the same antioxidant ability [29], and each phenolic compound contained in the latex extract can have different interactions during antioxidant assay [53].

## 4. Conclusion

The present study for the first time provides screening and identification of laticifers in vegetative organs of *Pergularia tomentosa*, including stem, leaf, and petiole. Anatomical studies revealed that the species is a nonarticulated laticifer type. By its functional group variety, latex composition was estimated as a complex of proteins, glucides, sterols, enzymes, lipids, etc. Rubber mainly contains *cis-*1-4-isoprene monomer as a major component.

From the above results, it can be concluded that the latex extract is a promising natural source of total phenolics and flavonoids. The low IC_50_ confirmed a higher ability to scavenge DPPH, and therefore, latex has an interesting antioxidant activity. The correlation between secondary metabolites and antioxidant activity of *Pergularia tomentosa* latex encourages researchers to prove the same therapeutic properties revealed with roots, leaves, stems, and fruit extracts mainly including antifungal, antimicrobial, antimolluscicidal, antiapoptic, and anti-inflammatory activities. The latex is often searched for industry application as protective gloves, shoes, and hoses and for medical equipment like gloves, tubing, and straps. The described properties led to more study and investigate the composition in order to its valorisation as a natural and an eco-friendly extract with a low cost.

## Figures and Tables

**Figure 1:** Photographs of latex exudation from vegetative aerial parts of *Pergularia tomentosa*. (a) Profuse latex exudation in stem (GX 10). (b) Latex exudation in stem (GX 10). (c) Detail of laticifers at stem level (GX 40). (d) Profuse latex exudation in petiole (GX 10). (e) Sectioned leaf showing latex droplets (GX 0).

**Figure 2:** Stem cross sections of *Pergularia tomentosa*. Fixation FAA, double staining (aceto-carmin). (a) Overview of fresh stem transverse section (GX 40). C: cortex; Cc: central cylinder. (b) Details of (a), showing the anatomical structure of the stem (GX 120). Pi: pith; Nt: nonglandular trichome; Ec: epiderm with thick cuticule; F: fiber; Cp: cortical parenchyma; Co: collenchyma; X: xylem II; P: phloem; L: laticifer.(c) Details of (b) (rectangle), high magnification of a laticifer (GX 1000).

**Figure 3:** Cross sections of leaf and petiole of *Pergularia*, stained with aceto-carmin and fixed with FAA. (a) Transverse sections at the midrib level of a leaf (GX 40). (b) Details of (a) (rectangle) showing laticifer (GX 100). Co: collenchyma; Le: lower epidermis; P: phloem; Sp: spongy parenchyma; Pp: palisade parenchyma; Ue: upper epidermis; X: xylem; L: laticifer; Nt: nonglandular trichome. (c) Overview of cross section of *Pergularia* petiole (GX 40). (d) Details of (c) (rectangle) showing laticifers (GX 120). Co: collenchyma; Cp: cortical parenchyma, Ph: phloem; X: xylem; L: laticifer; Nt: nonglandular trichome.

**Figure 4:** FTIR spectra of *Pergularia tomentosa* latex extract.

## Data Availability

The data is available upon request.
